The article "Application of Neural Network Algorithm Combined with Bee Colony Algorithm in English Course Recommendation" was retracted in 2023. Reasons: unreliable results or conclusions; concerns about the data; concerns about the peer review; concerns about the citations.

# Application of Neural Network Algorithm Combined with Bee Colony Algorithm in English Course Recommendation

**DOI:** 10.1155/2021/5307646

**Published:** 2021-12-20

**Authors:** Guiting Ren

**Affiliations:** School of Humanities, Shangluo University, Shangluo 726000, Shaanxi, China

## Abstract

The traditional BP neural network has the disadvantages of easy falling into local minimum and slow convergence speed. Aiming at the shortcomings of BP neural network (BP neural network), an artificial bee colony algorithm (ABC) is proposed to cross-optimize the weight and threshold of BP network parameters. This study is mainly about the application of BP neural network algorithm in English curriculum recommendation technology. It includes the application of BP neural network algorithm in English course recommendation technology, English course teaching design mode, the application of BP neural network algorithm in English course, and the optimal combination of bee colony algorithm and BP neural network. After 4690 iterations, the neural network reaches the target accuracy, and the training is completed. At the same time, the prediction error of the model is less than 10%, which further shows that the performance of the prediction model is good. Therefore, the combination model is recommended in this paper. The results show that the optimization algorithm improves the solution accuracy and speeds up the convergence speed of the network.

## 1. Introduction

Optimization technology is an application technology based on mathematics to find the best feasible solution for a target optimization problem under certain time constraints [1]. The calculus proposed in the seventeenth century contained the idea of optimization. The self-optimization theory has been put forward, and its research has always been very active, and with the development of science and technology, people's research on optimization technology has become more and more in-depth, which has also played an important role in promoting the development of human civilization [2]. The Chinese English Curriculum Standard (experimental draft) formulated by the Ministry of education of China was officially published in 2001. This curriculum standard embodies a new educational concept, determines the nature and task of the new English curriculum, describes the specific curriculum objectives and contents, and puts forward specific implementation suggestions. As a guiding principle, this curriculum standard will have a great and profound impact on the reform of English education in China [3].

Machine learning (ML) is an important research field of artificial intelligence and computer science and has gradually developed into an important technical support of other related disciplines. Especially, in recent years, there are constantly adopting-driven machine learning methods, and data analysis technology using machine learning has become one of the important technologies to solve complex problems [4]. Artificial bee colony algorithm is an optimization algorithm proposed based on the behavior of individuals in the bee colony to search for pollen in cooperation with each other. It has a strong global search performance. Although the research and application of Bee Colony Algorithm (BP) have not been long, more and more scholars have studied it due to the advantages of fewer parameters and easy implementation [5].

The article "Application of Neural Network Algorithm Combined with Bee Colony Algorithm in English Course Recommendation" was retracted in 2023. Reasons: unreliable results or conclusions; concerns about the data; concerns about the peer review; concerns about the citations.

In 2009, Karaboga and others completed the training of neural network by ABC algorithm and achieved good results [6]. As an advanced artificial intelligence technology, Neural Network Algorithm is very suitable for dealing with nonlinear and noisy data, especially for those problems characterized by fuzzy, incomplete, and incomplete knowledge or data [7]. Neural network algorithm has the advantages of self-adaptation, self-learning, self-organization, good fault tolerance, robustness, parallelism, and associative memory and has been widely used to solve the problems of pattern recognition, prediction, optimization control, and intelligent decision-making [8]. The curriculum design of “Standard” proposes to set up compulsory courses and elective courses, design courses based on “study field-subject-module,” and implement the credit system of curriculum management. Among the compulsory courses, there are comprehensive courses of English 1, 2, 3, 4, 5, and 6. Elective courses include English-Chinese translation, practical writing, newspaper reading, English speech, secretarial English, technical English, English literature appreciation, film and television appreciation courses. This is almost a copy of all the college English courses in most colleges and universities. If college English is not reformed, it will inevitably lead to great duplication and waste of teaching resources [9].

The traditional BP neural network has the disadvantages of easy falling into local minimum and slow convergence speed. Aiming at the shortcomings of traditional BP neural network (BP neural network), this paper creatively proposes an artificial bee colony algorithm (ABC) to cross-optimize the weight and threshold of BP network parameters. This study is mainly about the application of BP neural network algorithm in English curriculum recommendation technology. The optimization algorithm improves the solution accuracy and speeds up the convergence speed of the network.

This paper is divided into five parts. The first part expounds the research background of different optimization technologies, including neural network and machine learning. The second part expounds the research of relevant literature. The third part expounds the content of artificial bee colony algorithm (ABC), and the fourth part expounds the BP neural network algorithm. It includes the application of BP neural network algorithm in English course recommendation technology, English course teaching design mode, and BP neural network algorithm in English course and optimizes the combination of bee colony algorithm and BP neural network. Finally, the full text is summarized.

The article "Application of Neural Network Algorithm Combined with Bee Colony Algorithm in English Course Recommendation" was retracted in 2023. Reasons: unreliable results or conclusions; concerns about the data; concerns about the peer review; concerns about the citations.

## 2. Related Work

With the deepening of people's understanding of nature and the rapid development of biology, many scholars and experts observe and study biological groups and begin to imitate the swarm intelligence generated by the cooperation of simple individuals to design algorithms to solve the optimization problems of complex systems. ABC is a new intelligent heuristic algorithm, which was proposed by Hu et al. [10]. The algorithm comes from the research and Simulation of honeybee behavior. Chen et al. put forward the error Backpropagation (BP) algorithm of multilayer feedforward network in Parallel Distributed Processing, which became a major turning point in the revival of neural network algorithm research [11]. Babaeizadeh et al. pointed out that the research of neural network includes the basic theory of neural network, network learning algorithm, network model, and network application, among which the more popular is the research of neural network learning algorithm. Among them, the BP algorithm is the most basic and most popular supervised learning algorithm, which is relatively mature both in theory and in practical applications [12]. Xu and SrIvastava further proposed that we should focus on how to organize various learning machines and make them into a system when we know the advantages and disadvantages of different models, so as to solve specific problems. Some researchers use different learning machines such as nearest neighbor classifier, neural network algorithm, support vector machine, and decision tree to construct hybrid ensemble [13].

Jia et al. research shows that, to realize personalized recommendation, we mainly recommend different courses to different learners based on cluster analysis technology. In the network education platform, it is necessary to recommend different courses to learners [14]. According to the different degree of interest of learners in courses, the learners should be clustered and divided into different clusters, and then the learners who have the greatest similarity with the target learners should be found in the same cluster, and the learners' interest in different courses should be used to recommend courses to the target learners. In the excitation function, piecewise function is used as excitation function, or steepness factor is introduced. Wu et al., through research, proposed to adjust the excitation function, so that the sigmoid nonlinear function can avoid the BP neural network error caused by the extremely large or extremely small neuron input, and even the network failure convergence occurs [15].

The article "Application of Neural Network Algorithm Combined with Bee Colony Algorithm in English Course Recommendation" was retracted in 2023. Reasons: unreliable results or conclusions; concerns about the data; concerns about the peer review; concerns about the citations.

The research of literature [16] shows that the convergence speed of traditional BP neural network is slow, and it is easy to fall into local optimum. By introducing BP to adjust the connection weight and threshold of the network, the global search ability of the network is improved, the training time of the network is reduced, and the training accuracy of BP neural network is improved. He et al. point out that, after China's successful accession to the World Trade Organization (WTO) in 2001, foreign exchanges have expanded and penetrated into many fields such as politics, economy, culture, science and technology, and military affairs, and there is an increasing demand for compound talents who are proficient in majors and have strong foreign language skills in all walks of life, and the instrumental and applied features of foreign languages have become increasingly prominent [17]. Hu et al. show that English teaching refers to learning English as the goal, but social constructivism believes that language learning should also have educational value and should be conducive to the overall development of learners [18]. An anonymous researcher pointed out that the evaluation of English courses should be based on the objectives and requirements of the curriculum standards to achieve effective monitoring of the entire teaching process and results, which clarifies the role of evaluation and the relationship with the curriculum [19].

## 3. Artificial Bee Colony Algorithm (ABC)

Artificial bee colony algorithm (ABC) is a swarm intelligent optimization algorithm that simulates the honey collecting behavior of bees. It provides a new method to solve the global optimization problem in the field of science. Because it has the advantages of few control parameters, easy implementation, and simple calculation, it has been concerned by more and more researchers. Honeybee is a social insect. The behavior of a single individual is very simple, and the ability is weak, but the group composed of individuals shows strong coordination ability and survival ability [20]. Bee colony in nature can always find high-quality honey source with high efficiency and can adapt to the change of environment and obtain higher income [21]. Usually, most of the worker bees stay in the hive for “in-house work,” and only a few of them search for food sources around the hive randomly. Once favorable honey gathering places or new high-quality honey sources are discovered, they will become honey gathering bees and fly back to the hive to tell the worker bees who are “back-office” in the hive about the location of food and the distance information between the hive and the honey source by dancing in circles or “Figure 1” and also tell the type of food and the quality of honey source by the smell of pollen on their bodies, calling on everyone to gather honey [22]. The worker bees in the nest can not only judge the direction and distance of the nectar source by detecting the dance of the bees, but also evaluate the quality of the nectar source from the excitement of the dance [23]. The honey-gathering process of bees is similar to the process of searching for the optimal solution of the problem to be optimized in evolutionary computing. Honeybee honey collection is realized through communication, transformation, and cooperation among different roles. The process of bee colony to collect honey includes three basic parts and two basic behaviors. The three parts are honey source, hired bee, and nonhired bee. The two behaviors are recruiting and giving up a honey source for the honey source [24].

The article "Application of Neural Network Algorithm Combined with Bee Colony Algorithm in English Course Recommendation" was retracted in 2023. Reasons: unreliable results or conclusions; concerns about the data; concerns about the peer review; concerns about the citations.

The solution process of ABC is to use bee colony to find the optimal solution by using roulette method and greedy algorithm in the candidate solution set [25]. The basic idea of the algorithm is to divide the bees into three types after initialization: leading bees, following bees, and reconnaissance bees. Generally, the leading bees and following bees have the same number, each accounting for half of the total number of bees. The reconnaissance bees are transformed by abandoning the leading bees with poor solutions, and there are generally no reconnaissance bees during initialization [26]. After the algorithm is initialized, each leading bee will generate a set of random solutions within the range of the solution set, and then the leading bee will perform a local search within the neighborhood of this set of solutions, and when a new food source is found, the greedy algorithm will choose a more random solution. Good food sources (discard poor food sources) stage is called the lead bee search stage [27]. After the leading bee search stage, enter the following bee search stage. The latter bees will choose a better food source according to the food source information provided by the leading bees and the selection method of roulette and then conduct neighborhood search near the selected food source. When new food sources are discovered, greedy algorithm is also used to select better food sources. If the newly discovered food source is better, the bees below will inform the leading bees in the front to update the food source information [28]. In the follow-up bee search stage, food sources with higher fitness will gather more follow-up bees to collect honey. With the increase of neighborhood search times, these food sources will have more opportunities to achieve optimization. Because the algorithm may fall into the local optimal solution, which makes the algorithm stagnate, ABC introduces the role of reconnaissance bee. Once the algorithm stagnates, the scout bees will appear, and then randomly search for new food sources and transmit the information to the leader bees, thus ensuring the diversity of races. Through the iteration of the algorithm, the three bees cooperate with each other, and finally the algorithm converges to the global optimal solution.

The article "Application of Neural Network Algorithm Combined with Bee Colony Algorithm in English Course Recommendation" was retracted in 2023. Reasons: unreliable results or conclusions; concerns about the data; concerns about the peer review; concerns about the citations.

Formula (1) is the update formula for the food source position of the leading bee and the follower bee:

(1) $$\begin{array}{c} v_{ij}=x_{ij}+r_{ij}\left(x_{ij}-x_{kj}\right). \end{array}$$

*k* ∈ (1,2,…, SN), *j* ∈ (1,2,…, *d*) are given randomly, but *k* cNeural Network Algorithm is equal to *i* (k is a solution of the neighborhood of *i*). The random number of *r*_*ij*_ ∈ [−1,1], which controls the generation of neighborhood of *x*_*ij*_ neighborhood. As the search approaches the optimal solution, the range of neighborhood will become smaller and smaller.

ABC algorithm (follow the bees to choose which food source) is by leading the swing of bees to determine the amount of nectar of the food source, and according to the amount of nectar to choose which food source to collect nectar. The number of nectars is expressed by fitness value, and the selection probability *P*_*i*_ is determined by the following formula:

(2) $$\begin{array}{c} P_{i}=\frac{{\text{fit}}_{i}}{\sum_{j=1}^{SN}{\text{fit}}_{j}}. \end{array}$$

Among them, fit_*i*_ represents the fitness value of the ith solution (food source), and SN is the number of solutions.

In this ABC algorithm, an adjustable parameter “limit” is added to record the update times of the solution. If the quality of the solution is not improved in the periodic scheme shown by this parameter, it means that the solution falls into local optimization. At this time, the solution will be abandoned, and the corresponding leading bee will become a reconnaissance bee. Assuming that the abandoned solution is *x*_*i*_ and *j*∈(1, 2,…, *d*), the scout bees randomly generate a new solution instead of *x*_*i*_ by using the updated formula of formula (1).

(3) $$\begin{array}{c} x_{i}^{j}=x_{\min}^{j}+\text{rand}\left(0,1\right)\left(x_{\max}^{j}-x_{\min}^{j}\right). \end{array}$$

The above analysis shows that the ABC algorithm performs four selection processes: ① follow the global selection process of finding a better food source according to formula (2). ② The leading bee and the follower bee follow formula (1) to perform the neighborhood search partial selection process. ③ All artificial bees make judgments and comparisons between the new and old food sources and retain a better solution to the greedy selection process. ④ There is the random selection process of the detective bee discovering the food source according to formula (3).

The article "Application of Neural Network Algorithm Combined with Bee Colony Algorithm in English Course Recommendation" was retracted in 2023. Reasons: unreliable results or conclusions; concerns about the data; concerns about the peer review; concerns about the citations.

In ABC algorithm, the essence of Scout bee's behavior is to increase the diversity of population and avoid the algorithm falling into local optimum. The parameter “limit” controlling its behavior has a great impact on the algorithm performance. It is troublesome to debug the parameters. Improper setting will greatly reduce the algorithm performance. Other operations can be taken to achieve the same effect. For f1 and f2 tests, change the value of limit. In order to avoid the bad influence of random population on algorithm evaluation and ensure the initial population unchanged, get the change curve of fitness value with different values of limit and compare the algorithm performance, as shown in Figures 2 and 3. It can be seen from Figures 2 and 3 that when “limit = 10,” the fitness value in the later stage of the algorithm is almost unchanged, while when “limit = 500,” the fitness value changes greatly. That is to say, under different values of limit, the corresponding fitness values of each generation of the algorithm are quite different; that is, the performance of the algorithm has a great relationship with the value of limit.

### 3.1. BP Neural Network Algorithm

BP neural network algorithm is composed of many parallel interconnected neurons. A neuron can be connected to many other neurons; that is, it can have multiple inputs, but it has only one output [29]. Neuron is the most basic information processing unit of neural network algorithm and is an abstract mathematical model, mainly composed of the following three basic elements:

1. Connection between artificial neurons: that is to say, the connection weights of neural networks. The weights are positive and negative. The positive weights indicate intensification, and the negative weights indicate inhibition.
2. Adder: it is an input signal accumulator, which is used to calculate the accumulated sum of the corresponding weights of the input signal and the neuron. This operation is only a linear operation.
3. Activation function: also known as transfer function or excitation function, which is mainly used to limit the output value of neurons in the range of activating or inhibiting synapses, that is, to limit the output of neurons in a certain allowable range, which is usually a closed interval such as [−1, 1] or [0, 1].

The article "Application of Neural Network Algorithm Combined with Bee Colony Algorithm in English Course Recommendation" was retracted in 2023. Reasons: unreliable results or conclusions; concerns about the data; concerns about the peer review; concerns about the citations.

As shown in Figure 4, it is a typical neuron model. There are *n* input signals connected to neuron *i*, and *w*_*ij*_ represents the synaptic strength or connection weight of the j-th input to neuron *i*. *u*_*i*_ is the net input of neuron *i*, which is obtained by linear combination of input signals through an accumulator, *b*_*i*_ is the deviation of the neuron, and *v*_*i*_ is the value adjusted by the deviation, which is also called the local sensing area of the neuron. *f*(·) is the activation function, and *y*_*i*_ is the output of neuron *i*. The corresponding calculation formulas for each parameter are shown in formulas (4)–(6):

(4) $$\begin{array}{c} u_{i}=\sum_{j=1}^{n}w_{ij}x_{j}, \end{array}$$

(5) $$\begin{array}{c} v_{i}=u_{i}+b_{i}, \end{array}$$

(6) $$\begin{array}{c} y_{i}=f\left(v_{i}\right). \end{array}$$

Network topology is an important feature of neural networks. Neural network is composed of a large number of parallel distributed and widely interconnected neurons, so the difference of network structure is mainly due to the different connection between neurons. From the viewpoint of connection, there are two kinds: feedforward neural network and feedback neural network; the latter is also called recurrent network.

1. Feedforward neural network is a hierarchical network formed by neuron hierarchical organization, and its structure is shown in Figure 5. It can be seen from the figure that the information in the network can only be transmitted in one direction; that is to say, the information sent by neurons can only be transmitted from one layer to the next layer until the result is output. There is no information exchange between neurons in the same layer or between neurons in different layers. Feedforward network is composed of multilayers, in which the input layer and output layer are connected with the outside world, and other middle layers are called hidden layers, which can be one or more layers. Feedforward network includes multilayer perceptron network, CMAC network, and learning vector quantization network.
2. Feedback neural network: the output result of the feedback neural network can affect the input and change the weights. Therefore, the signal of the network can propagate in both positive and negative directions. The structure is shown in Figure 6. Hopfield network, Elman network, and Jordan network are more commonly used feedback neural networks.

The article "Application of Neural Network Algorithm Combined with Bee Colony Algorithm in English Course Recommendation" was retracted in 2023. Reasons: unreliable results or conclusions; concerns about the data; concerns about the peer review; concerns about the citations.

Figure 7 is the employment rate error curve of each algorithm based on the number of iterations. In the iterative training process of each algorithm, the network error presents a downward trend with the increase of the number of iterations. At the beginning, the decrease is particularly fast. After a period of iteration, it gradually tends to be flat and finally reaches the convergence state.

## 4. Application of BP Neural Network Algorithm in English Course Recommendation Technology

### 4.1. Teaching Design Model of English Course

The traditional view of education believes that learning is the acquisition of knowledge, while social constructivism believes that the ability is more important than knowledge. With the ability, you can acquire knowledge. Of course, knowledge is also an important basis for composing ability. In terms of name alone, the traditional syllabus has been changed to the current English curriculum standards. The syllabus refers to the description of the content and teaching sequence of a course, while the English curriculum standards also include the study of English curriculum settings, system objectives, implementation methods, and evaluation. The learner's evaluation of English courses can be explicit or implicit. Explicit evaluation usually means that learners rate an English course in numerical form. If the value is very high, it means that the learner likes the English course very much; otherwise, it means that the learner does not like the English course. This method requires a special questionnaire survey. If the learner wants to get the help of the recommendation system, he first needs to submit his evaluation information of some English courses to the system. Implicit evaluation is usually derived from data resources. It is generally believed that the instructional design is based on system theory, learning theory, and communication theory, using systematic methods to analyze teaching problems, determine teaching goals, and establish strategies to solve teaching problems Plan, trial solution, evaluate trial results, and modify plan to get an optimized teaching process.

Since the end of 1960s, the research on instructional design has made great progress. According to the statistics of Andrews and Goodson in 1980, there were only 40 ID models in the literature at that time, and the number increased to hundreds in 1991. Although people from different angles of teaching system have different understanding of teaching design. But almost any instructional design has the same goal: to help optimize teaching. This is mainly reflected in the following aspects: instructional design can make teaching objectives clear and comprehensive and provide teachers with a psychological reference framework in the implementation of teaching activities, so as to achieve teaching objectives practically. Instructional design can guide teachers to choose effective teaching methods and arrange teaching activities according to teaching objectives, learners' characteristics, and the nature of learning content. Instructional design helps educational practitioners allocate teaching time according to the specific situation of teaching process and improve teaching efficiency.

The article "Application of Neural Network Algorithm Combined with Bee Colony Algorithm in English Course Recommendation" was retracted in 2023. Reasons: unreliable results or conclusions; concerns about the data; concerns about the peer review; concerns about the citations.

### 4.2. BP Neural Network Algorithms in English Course

In the actual neural network, there is a phenomenon of lateral inhibition that is, after a nerve cell is excited, its branches will inhibit other surrounding nerve cells. This inhibition causes competition between nerve cells and the one with the strongest excitement. The nerve cells of nerve also strongly inhibit peripheral nerve cells. Although each nerve cell is in a state of excitement at the beginning, in the end, the nerve cell with the largest output “wins,” and the surrounding nerve cells “lose.”

In addition, in the cognitive process, in addition to getting knowledge from teachers, there is also a kind of learning that does not need teachers' guidance. For example, after a baby is born, when he hears the stimulation of external sound, he will naturally make a sound and learn to grasp things and walk in the external environment. This phenomenon is more common in animals. This kind of function, which directly depends on external stimulation, is sometimes called self-learning and self-organizing learning method. Traditional English teaching cannot pay enough attention to the differences of each student and cannot provide a more perfect service system. This paper mainly analyzes the BP neural network as the algorithm, focusing on the basic principle of BP algorithm, the specific steps of training, and the heuristic rules of evaluation application. The final results show that English teaching can meet the needs of students and has good stability.

Self-organizing feature map (SOM) neural network algorithm is generated based on the above two biological structures and phenomena. Network training is mainly based on the cross-correlation between adjacent node excitations, so it can organize itself without external supervision. The output units compete with each other, and finally only the strongest one wins and is activated to suppress the output of other units. Output arrangement forms an ordered topological image, which reflects the similarity between input signals.

The article "Application of Neural Network Algorithm Combined with Bee Colony Algorithm in English Course Recommendation" was retracted in 2023. Reasons: unreliable results or conclusions; concerns about the data; concerns about the peer review; concerns about the citations.

Suppose that the sample observation set {*X*_1_, *X*_2_,…, *X*_*p*_} is composed of n-dimensional real vectors, namely, *X*_*j*_=[*x*_*j*1_, *x*_*j*2_,…, *x*_*jn*_]. The ith output node is denoted as *m*_*i*_, and the connection weights between each output node and *n* input nodes constitute an n-dimensional vector, which is called a node vector and is also denoted as *m*_*i*_, *m*_*i*_(*t*)=[*m*_*i*1_(*t*), *m*_*i*2_(*t*),…, *m*_*in*_(*t*)], where *t* is the number of learning.

The general SOM algorithm can be described as follows:

(1) In the observation sample set {*X*_1_, *X*_2_,…, *X*_*p*_}, a *X*_*j*_ input network is randomly selected.
(2) The winning node *m*_*c*_(*t*) is selected according to the principle of minimum distance $\left\|X_{j}-m_{c}\left(t\right)\right\|=\underset{t}{\min}\left\|X_{j}-m_{i}\left(t\right)\right\|$, where ‖·‖ can be defined as Euclidean distance. At this time, the node *m*_*c*_ can be called *X*_*j*_ activated.
(3) Adjust the connection weight vector *m*_*i*_(*t*) : *m*_*i*_(*t*+1)=*m*_*i*_(*t*)+*T*(*t*) · *h*_*ci*_(*t*)[*X*_*j*_ − *m*_*i*_(*t*)]. *T* (*t*) is a learning rate factor, which is selected as a decreasing function of learning times *t* in order to make the algorithm converge. *h*_*ci*_(*t*) is called neighborhood function. After it is introduced, the algorithm adjusts not only the winning node vector, but also the nearby nodes in each step, so the distance between nodes and input data in this area is closer than before. At the end of learning, the activated nodes of two similar input data are closer, so the topological relationship of input data is well preserved on the output plane. If the output node is represented by the point *r*_*i*_ in the two-dimensional space, *h*_*ci*_(*t*)=exp[−‖*r*_*c*_ − *r*_*i*_‖^2^/2^*e*^(*t*)^2^] can be defined, where *r*_*c*_ represents the winning node, and ^*e*^(*t*) is a monotonically decreasing function with the number of learning times *T*, such as a linear function that tends to zero, so when learning is over, it degenerates into
  (7) $$\begin{array}{c} h_{ci}\left\{\begin{array}{cc} 1, & i=c,\\ 0, & i\neq c. \end{array}\right) \end{array}$$
(4) From this, the variational equation describing the change of the node *m*_*i*_(*t*) vector can be obtained:

(8) $$\begin{array}{c} \Delta m_{i}\left(t\right)=T\left(t\right)h_{ci}\cdot \left(X_{j}-m_{i}\left(t\right)\right). \end{array}$$

When reaching a steady state, there is *E*[*h*_*ci*_(*t*) · (*X* − *m*_*i*_^*∗*^)]=0, where *m*_*i*_^*∗*^ is the stable convergence value of mi (*t*). By the nature of *h*_*ci*_(*t*), at the end of the study, $h_{ci}\left\{\begin{array}{cc} 1, & i=c,\\ 0, & i\neq c \end{array}\right)$. Let *V*_*i*_ be the set of all nodes that activate *m*_*i*_^*∗*^, *numb*(*V*_*i*_) represents the number of elements in Vi, *numb*(*V*_*i*_) is relatively large at first, and then it decreases with the increase of the number of learning. Based on the above analysis, the following self-organizing learning algorithm in batch processing can be obtained:

- Determine the number of input nodes, output nodes, and the initial value of node vector (MI = mi (0) is a small random quantity).
- Input all data into the network one by one, and adjust each node vector *m*_*i*_(*t*) to make *m*_*i*_(*t*+1)=∑_*j*∈*V*_*i*__*X*_*j*_/*numb*(*V*_*i*_). Learning is repeated until the excited neurons on the output neuron plane correspond to the input samples stably.

The article "Application of Neural Network Algorithm Combined with Bee Colony Algorithm in English Course Recommendation" was retracted in 2023. Reasons: unreliable results or conclusions; concerns about the data; concerns about the peer review; concerns about the citations.

The main reason for choosing BP neural network is that, compared with single-layer networks such as Least mean square and Levenberg-Marquardt, BP neural network is a multilayer network and has better nonlinear fitting capabilities. As shown in Figure 8, after 4690 iterations, the neural network reaches the target accuracy, and training is complete.

### 4.3. Combination of Optimized Bee Colony Algorithm and BP Neural Network

Chemical mechanical polishing (CMP) was developed by IBM in the 1980s. It is a processing technology combining mechanical grinding and chemical dissolution, which avoids the disadvantages of simple chemical grinding, slow speed, poor consistency, and easy to cause surface damage. This is the only technology that can realize the global flattening of multilayer copper wire. BP neural network based on optimized bee colony algorithm inherits the structure of traditional BP neural network. By introducing swarm intelligence algorithm, the global search ability of BP neural network is improved, the convergence speed of BP neural network is improved, and the possibility of falling into local optimal solution is reduced. A CMP polishing rate prediction model is established by combining bee colony algorithm and BP neural network. The prediction results of the model are shown in Figures 1 and 9. It can be seen from Figure 1 that, from the prediction of several groups of data, the model has good prediction ability, can more accurately simulate the polishing rate of CMP, and can establish more accurate polishing temperature. The composition of polishing solution and polishing solution can be seen in Figure 9 where the prediction error of the model is within 10%, which further indicates the better performance of the prediction model.

Because of this combination, the model has good prediction ability, can more accurately simulate the polishing rate of CMP, and can establish a more accurate polishing temperature. At the same time, the prediction error of the model is less than 10%, which further shows that the performance of the prediction model is better. Therefore, the combination model is recommended in this paper.

The article "Application of Neural Network Algorithm Combined with Bee Colony Algorithm in English Course Recommendation" was retracted in 2023. Reasons: unreliable results or conclusions; concerns about the data; concerns about the peer review; concerns about the citations.

## 5. Conclusions

In view of the shortcomings of neural network learning algorithm, the evolutionary method is combined with network training; that is, ABC method is used to optimize the mean square error function of the network, so as to obtain the optimal weight and threshold of the network. By introducing swarm intelligence algorithm, the global search ability of BP neural network is improved, the convergence speed of BP neural network is improved, and the possibility of falling into local optimal solution is reduced. A CMP polishing rate prediction model is established by combining bee colony algorithm with BP neural network. The prediction results of the model are shown in Figures 1 and 9. It can be seen from the test that, from the prediction of several groups of data, the model has good prediction ability, can more accurately simulate the polishing rate of CMP, and can establish a more accurate polishing temperature. At the same time, the model error is less than 10%, which further shows the high accuracy. Compared with the traditional BP neural network, the algorithm is not easy to fall into local minimum, and the convergence speed is slow. Compared with other intelligent algorithms, BP algorithm has some advantages, but it also has some limitations. Future research will position English Curriculum in an open system to make it close to reality, life, and the times. Developing English curriculum resources, using teaching materials flexibly, and adjusting teaching methods can achieve teaching objectives more effectively.

## Figures and Tables

**Figure 1:** Comparison of predicted value and measured value of CMP polishing rate prediction model.

**Figure 2:** The test effect of each algorithm on f1.

**Figure 3:** The test effect of each algorithm on f2.

**Figure 4:** Neuron model.

**Figure 5:** Feedforward neural network.

**Figure 6:** Feedback neural network.

**Figure 7:** Error curve.

**Figure 8:** The BP neural network reached the preset accuracy after 4690 iterations.

**Figure 9:** The prediction error of the CMP polishing rate prediction model.

## Data Availability

The data used to support the findings of this study are available upon request to the author.
